# Circular RNA circPVT1 Contributes to Doxorubicin (DXR) Resistance of Osteosarcoma Cells by Regulating TRIAP1 via miR-137

**DOI:** 10.1155/2021/7463867

**Published:** 2021-04-23

**Authors:** Dan Li, Yan Huang, Gang Wang

**Affiliations:** ^1^Department of Radiology, The First Hospital of Jilin University, Changchun City, Jilin Province, China; ^2^Department of Orthopedics, China-Japan Union Hospital of Jilin University, Changchun City, Jilin Province, China

## Abstract

**Background:**

Chemoresistance is a major obstacle to the treatment of osteosarcoma patients. Circular RNA (circRNA) circPVT1 has been reported to be related to the doxorubicin (DXR) resistance in osteosarcoma. This study is designed to explore the role and mechanism of circPVT1 in the DXR resistance of osteosarcoma.

**Methods:**

circPVT1, microRNA-137 (miR-137), and TP53-regulated inhibitor of apoptosis 1 (TRIAP1) levels were detected by real-time quantitative polymerase chain reaction (RT-qPCR). The protein levels of ATP-binding cassette, subfamily C, member 1 (ABCC1), multidrug resistance-associated protein 1 (MRP-1), cleaved- (c-) caspase-3, B-cell lymphoma-2 (Bcl-2), and TRIAP1 were examined by a western blot assay. Cell viability, proliferation, and apoptosis were detected by cell counting kit-8 (CCK-8), colony formation, and flow cytometry assays, severally. The binding relationship between miR-137 and circPVT1 or TRIAP1 was predicted by starbase 3.0 and then verified by dual-luciferase reporter and RNA Immunoprecipitation (RIP) assays. The biological role of circPVT1 in osteosarcoma tumor growth and drug resistance was examined by the xenograft tumor model *in vivo. Results*. circPVT1 and TRIAP1 were highly expressed, and miR-137 was decreased in DXR-resistant osteosarcoma tissues and cells. Moreover, circPVT1 knockdown could boost DXR sensitivity by inhibiting DXR-caused proliferation and DXR-induced apoptosis in DXR-resistant osteosarcoma cells *in vitro*. The mechanical analysis discovered that circPVT1 acted as a sponge of miR-137 to regulate TRIAP1 expression. circPVT1 silencing increased the drug sensitivity of osteosarcoma *in vivo. Conclusion*. circPVT1 boosted DXR resistance of osteosarcoma cells partly by regulating the miR-137/TRIAP1 axis, hinting a promising therapeutic target for the osteosarcoma treatment.

## 1. Introduction

Osteosarcoma, which occurs mainly in children and adolescents, is the most common malignant bone tumor [1, 2]. Despite substantial progress in detection and therapeutic methods, the prognosis of osteosarcoma patients remains poor [3, 4]. Notably, chemotherapy has been considered to improve survival and reduce symptoms of osteosarcoma, but treatment failure often occurs owing to intrinsic or acquired chemoresistance [5]. Hence, it is imperative to find the underlying molecular mechanism of chemoresistance in osteosarcoma.

As a novel class of noncoding RNAs, circular RNAs (circRNAs) are characterized by a covalently closed loop without 5′ caps and 3′ polyadenylated tail [6]. circRNAs are widely expressed in mammalian cells and have been reported to regulate gene expression at different levels [7]. An extensive body of research indicated that the dysregulation of circRNAs participated in the development and progression of diverse cancers, serving as oncogenes or tumor suppressors [8, 9]. Furthermore, circRNAs have been reported to be closely related to chemoresistance in a variety of cancers, including osteosarcoma. For example, Dong and Qu showed that circRNA circUBAP2 boosted the cisplatin resistance in osteosarcoma through regulating the miR-506-3p-mediated Wnt/*β*-catenin signaling pathway [10]. circPVT1, transcribed from the long noncoding RNA region with PVT1 locus on chromosome 8q24, has been confirmed to promote chemotherapy resistance in some cancers [11, 12]. Moreover, circPVT1 was presented to be increased in osteosarcoma and facilitated the doxorubicin (DXR) resistance of osteosarcoma cells [13, 14]. Unfortunately, the exact mechanism of circPVT1 in DXR resistance of osteosarcoma has not been fully clarified.

Small endogenous noncoding RNA, microRNAs (miRNAs), could take part in the regulation of gene expression at the posttranscriptional level [15]. Several reports have exhibited that the abnormal expression of miRNAs is associated with drug resistance in many types of cancer, including osteosarcoma [16–18]. MicroRNA-137 (miR-137) displayed abnormally low expression in human cancers, such as lung cancer [19], hepatocellular carcinoma [20], and osteosarcoma [21]. Importantly, the relevant literature reported that miR-137 was decreased in DXR-resistant osteosarcoma cell lines, and the overexpression of miR-137 could weaken the DXR resistance of osteosarcoma cells [22], suggesting the pivotal role of miR-137 in DXR resistance in osteosarcoma.

TP53-regulated inhibitor of apoptosis 1 (TRIAP1), an apoptosis inhibitor, has been identified as a novel effector of drug resistance in various cancers [23]. For instance, the downregulation of TRIAP1 could enhance the cisplatin sensitivity in human ovarian cancer by activating the cytochrome c/Apaf-1/caspase-9 pathway [24]. Also, TRIAP1, as a target of miR-107, was connected with the regulation of taxol sensitivity of breast cancer [25]. In osteosarcoma cells, TRIAP1 was increased and participated in the epirubicin-mediated antiproliferation and proapoptosis [26]. However, the role of TRIAP1 in DXR resistance in osteosarcoma is still largely unknown.

Here, circPVT1 was upregulated in DXR-resistant osteosarcoma cells and contributed to the DXR resistance in osteosarcoma. Using the bioinformatic analysis, there was the latent binding between miR-137 and circPVT1 or TRIAP1. Thus, the purpose of this study was to prove the role of circPVT1 and to explore whether the involvement of circPVT1 on DXR resistance in osteosarcoma was regulated by the miR-137/TRIAP1 axis.

## 2. Materials and Methods

### 2.1. Clinical Samples and Cell Culture

Osteosarcoma tissue samples were collected from 52 patients diagnosed with osteosarcoma at The First Hospital of Jilin University, and 45 normal bone tissue samples were provided by the volunteers from The First Hospital of Jilin University. Then, 52 osteosarcoma patients were divided into the chemoresistant group (*n* = 21) who showed <90% tumor necrosis after chemotherapy and the chemosensitive group (*n* = 31) who presented ≥90% tumor necrosis after chemotherapy, in line with the previous description [27]. This research got approved by the Ethics Committee of The First Hospital of Jilin University, and written informed consent was provided by every participant.

The human fetal osteoblastic cell line (hFOB1.19), human osteosarcoma cell lines (KHOS and U2OS), and 293T cell line were purchased from American Type Culture Collection (ATCC, Manassas, VA, USA). Under the humidified air atmosphere containing 5% CO_2_ at 37°C, cells were cultured in Dulbecco's modified Eagle's medium (DMEM; Gibco, Carlsbad, CA, USA) with 10% fetal bovine serum (FBS; Gibco) and 1% penicillin/streptomycin (Invitrogen, Carlsbad, CA, USA). Besides, DXR-resistant osteosarcoma cells (KHOS/DXR and U2OS/DXR) were established as previously [28], and the established cells were kept in the conditioned medium with 1 *μ*g/mL DXR (Sigma-Aldrich, St. Louis, MO, USA) to maintain their drug-resistant phenotype.

### 2.2. Real-Time Quantitative Polymerase Chain Reaction (RT-qPCR)

According to the standard protocol, total RNA from tissues and cells was first extracted by using the TRIzol reagent (Invitrogen). After quantification with NanoDrop (NanoDrop Technologies, Wilmington, WI, USA), the extracted RNAs were reverse-transcribed to the first-strand complementary DNA (cDNA) using the PrimeScript™ RT Master Mix (TaKaRa, Dalian, China). With the help of the Thermal Cycler CFX6 System (Bio-Rad, California, USA), RT-qPCR was carried out using an SYBR Green PCR Kit (TaKaRa). Then, the obtained data were calculated by the 2^–*ΔΔ*Ct^ method, normalized to glyceraldehyde 3-phosphate dehydrogenase (GAPDH for circPVT1 and TRIAP1) and U6 (for miR-137). The primers are showed in Table 1.

### 2.3. Western Blot Assay

In brief, RIPA buffer including a protease inhibitor (Beyotime, Nantong, China) was applied to harvest the protein lysates from tissues or cells, followed by quantification with the Pierce™ BCA Protein Assay Kit (ThermoFisher Scientific, Rockford, IL, USA). And then, protein samples (50 *μ*g) were separated with a sodium dodecyl sulfate-polyacrylamide gel electrophoresis (SDS-PAGE) system, which was further transferred onto nitrocellulose membranes (Millipore, New York, NY, USA). After blocking in 5% nonfat milk for 2 h, the membrane was incubated with primary antibodies against ATP-binding cassette, subfamily C, member 1 (ABCC1, 1 : 1000, ab170904, Abcam, Cambridge, MA, USA), multidrug resistance-associated protein 1 (MRP-1, 1 : 1000, ab9531, Abcam), cleaved- (c-) caspase-3 (1 : 1000, ab2302, Abcam), B-cell lymphoma-2 (Bcl-2, 1 : 1000, ab59348, Abcam), TRIAP1 (1 : 1000, ab225938, Abcam), and GAPDH (1 : 1000, ab9485, Abcam) at 4°C overnight. The next day, the membranes were probed with the corresponding secondary antibodies for 1 h, and the protein bands were detected according to the enhanced chemiluminescence reagent (ECL; GE Healthcare, Piscataway, NJ, USA).

### 2.4. Cell Transfection

In this assay, circPVT1 small interfering RNA (si-circ) and scrambled siRNA control (si-NC), miR-137 mimic, miR-137 inhibitor, and their negative controls (mimic NC and inhibitor NC) were obtained from RiboBio (Guangzhou, China). Moreover, the sequence of TRIAP1 was subcloned into pcDNA vector (Invitrogen) to obtain the pcDNA-TRIAP1 overexpression plasmid (oe-TRIAP1), and the pcDNA empty vector (Invitrogen) acted as the corresponding control (vector). Finally, all transfection of KHOS/DXR and U2OS/DXR cells was conducted referring to the instructions of the Lipofectamine 3000 reagent (Invitrogen).

### 2.5. Drug Resistance Assay

Generally, after 48 h of transfection in 96-well plates, KHOS/DXR and U2OS/DXR cells (5 × 10^3^ cells/well) were treated with different concentrations of DXR (0, 2, 4, 8, 16, 32, and 64 *μ*g/mL) for 48 h. Then, 10 *μ*L cell counting kit-8 (CCK-8, Dojindo, Kumamoto, Japan) solution was added into each well for 4 h, and the optical density was assessed with a microplate reader (TECAN M1000, Austria GmbH, Austria) at a wavelength of 450 nm. The relative survival curve was used to exhibit the concentration of DXR triggering 50% inhibition of growth (IC50).

### 2.6. Colony Formation Assay

In this assay, transfected KHOS/DXR and U2OS/DXR cells in 6-well plates were incubated with DXR (8 *μ*g/mL) for two weeks, followed by discarding the medium. After washing with phosphate-buffered saline (PBS, Invitrogen), the numbers of colonies per well were fixed 4% for 30 min and stained with 0.1% crystal violet. At last, visible colonies were imaged and counted manually.

### 2.7. Cell Apoptosis Assay

Transfected KHOS/DXR and U2OS/DXR cells were treated with 8 *μ*g/mL DXR for 48 h, followed by washing with PBS (Invitrogen). Then, the treated cells were stained with 5 *μ*L of Annexin (V-fluorescein isothiocyanate) V-FITC/Propidium Iodide (PI) (Selleck, Shanghai, China). According to FACSan flow cytometry (BD Biosciences, San Jose, CA, USA), the stained cells were examined, followed by analysis with Cell Quest software (BD Biosciences, Franklin Lakes, NJ, USA).

### 2.8. Dual-Luciferase Reporter Assay

Using the starbase 3.0 software, the potential relationship between miR-137 and circPVT1 or TRIAP1 was predicted. Then, the dual-luciferase reporter assay was applied to verify the consequence in 293T cells. Briefly, the sequences of circPVT1 and TRIAP1 3′-untranslated region (3′UTR) harboring wild-type (wt) or mutant-type (mut) putative miR-137 binding sites were amplified and inserted into pmirGLO vector (Promega, Madison, Wisconsin, USA), namely, circPVT1 wt/mut and TRIAP1 3′UTR wt/mut reporter vectors. And then, the constructed reporter vectors and miR-137 mimic or mimic NC were cotransfected into the 293T cells, following the operation manual of the Lipofectamine 3000 reagent (Invitrogen). After incubation for 48 h, a dual-luciferase reporter assay kit (Beckman Coulter, Fullerton, CA, USA) was employed to analyze the luciferase activities.

### 2.9. RNA Immunoprecipitation (RIP)

In this assay, the RIP assay was conducted using the Magna RIP RNA-binding protein immunoprecipitation kit (Millipore, Billerica, MA, USA). After treating with RIP lysis buffer, KHOS/DXR and U2OS/DXR cells were incubated with the magnetic beads conjugated with anti-Argonaute2 (Ago2) antibody or negative control IgG. After 6 h of incubation, the proteinase K was utilized to digest the samples, and coprecipitated RNA was segregated. The purified RNA was analyzed by using RT-qPCR.

### 2.10. Tumor Xenograft Assay

Our study got approved by the Animal Ethics Committee of The First Hospital of Jilin University. At first, circPVT1 knockdown stable lentiviral vector (lenti-short hairpin-circPVT1, termed as sh-circ) and the corresponding control (sh-NC) were provided by GeneChem (Shanghai, China). BALB/C nude mice (male, 3–4 weeks old, *n* = 6 per group) were gained from Vital River Laboratory (Beijing, China). Then, KHOS/DXR cells (5 × 10^6^) stably transfected with sh-circ or sh-NC were subcutaneously injected into the nude mice. At the indicated time points (7, 14, 21, 28, and 35 days), tumor volume was measured. At 35 days upon cell inoculation, the mice were sacrificed, and the tumors were excised and weighed.

### 2.11. Statistical Analysis

All data were analyzed with GraphPad Prism7 software. Pearson correlation analysis was used to analyze the expression association between miR-137 and circPVT1 or TRIAP1. Student's *t*-test or one-way analysis of variance (ANOVA) with Tukey's tests was used for the comparisons between two groups or multiple groups. Data of three independent experiments were shown as the mean ± standard deviation (SD). When *P* value < 0.05, it was considered to be statistically significant.

## 3. Results

### 3.1. circPVT1 Expression Was Upregulated in Osteosarcoma Tissues and Cells

Firstly, to investigate the function of circPVT1 in osteosarcoma, its expression level was examined in osteosarcoma tissues. Results showed that circPVT1 was increased in 52 osteosarcoma tissues relative to 45 normal tissues (Figure 1(a)). Then, according to the clinical information, 52 osteosarcoma patients were divided into the chemosensitive group (*n* = 31) and the chemoresistant group (*n* = 21). Our data suggested that the expression of circPVT1 was apparently higher in the chemoresistant group compared with the chemosensitive group (Figure 1(b)). Given the well-known roles of ABCB1 and MRP-1 in multidrug resistance, their expression levels were detected in osteosarcoma by a western blot assay. As displayed in Figures 1(c) and 1(d), the significant upregulation of ABCB1 and MRP-1 was viewed in osteosarcoma tissues and the chemoresistant group when compared with their respective control groups. Moreover, we further verified that circPVT1 was expressed at a high level in DXR-resistant osteosarcoma cells (KHOS/DXR and U2OS/DXR) versus parental osteosarcoma cells (KHOS and U2OS) and human fetal osteoblastic cell line (hFOB1.19) (Figure 1(e)). Meanwhile, our data suggested that the protein levels of ABCB1 and MRP-1 were increased in DXR-resistant osteosarcoma cells (KHOS/DXR and U2OS/DXR) in comparison with parental osteosarcoma cells (KHOS and U2OS) (Figure 1(f)). In a word, the dysregulation of circPVT1 might be associated with DXR resistance in osteosarcoma.

### 3.2. circPVT1 Knockdown Improved DXR Sensitivity in DXR-Resistant Osteosarcoma Cells

Considering the higher expression of circPVT1 in KHOS/DXR and U2OS/DXR cells, we knocked down circPVT1 in those cell lines. As shown in Figure 2(a), the expression level of circPVT1 was markedly decreased in si-circ-transfected KHOS/DXR and U2OS/DXR cells compared to cells transfected with si-NC. Then, we used the knocking down systems to further identify the effects of circPVT1 on DXR resistance in osteosarcoma cells. At first, transfected cells were treated with various concentrations of DXR for 48 h, and then, the IC50 value was detected by the CCK-8 assay. Results suggested that the IC50 value of DXR in KHOS/DXR and U2OS/DXR cells transfected with si-circ was lower than that in cells transfected with si-NC (Figure 2(b)). Moreover, the cell colony formation and flow cytometry assays indicated that circPVT1 knockdown led to a substantial decline in the clone number and a striking increase in the apoptosis rate in KHOS/DXR and U2OS/DXR cells (Figures 2(c) and 2(d)). To further verify the role of circPVT1 in DXR resistance in osteosarcoma cells, the apoptosis-related proteins (antiapoptotic factor: Bcl-2 and proapoptotic factor: c-caspase-3) and multidrug-resistant proteins (ABCB1 and MRP-1) were detected in KHOS/DXR and U2OS/DXR cells. As expected, the decreased protein levels of Bcl-2, ABCB1, and MRP-1 and increased c-caspase-3 levels were observed caused by the silencing of circPVT1 in KHOS/DXR and U2OS/DXR cells (Figure 2(e)). These data manifested that circPVT1 depletion sensitized KHOS/DXR and U2OS/DXR cells to DXR.

### 3.3. miR-137 Acted as a Target of circPVT1

Previous studies have presented that miR-137 worked as a tumor suppressor in osteosarcoma [29]. Thus, we detected the expression level of miR-137 in osteosarcoma tissues by the RT-qPCR assay. Data exhibited that miR-137 was reduced in osteosarcoma tissues (*n* = 52) compared with normal tissues (*n* = 45) (Figure 3(a)). More importantly, we found a significant decrease of miR-137 in the chemoresistant group and DXR-resistant osteosarcoma cells (KHOS/DXR and U2OS/DXR) (Figures 3(b) and 3(c)), implying the involvement of miR-137 in DXR resistance in osteosarcoma cells. Moreover, the miR-137 expression level was inversely correlated with the circPVT1 level in osteosarcoma cells (Figure 3(d)). Therefore, we explored the relationship between miR-137 and circPVT1 by using starbase 3.0. As presented in Figure 3(e), there were some complementary sites between circPVT1 and miR-137. To confirm the prediction, a dual-luciferase reporter assay was conducted in 293T cells. Data suggested that miR-137 mimic declined the luciferase activity of circPVT1 wt reporter vector but had no apparent impact on luciferase activity of circPVT1 mut reporter vector (Figure 3(f)). Then, to further validate the mutual effect of circPVT1 and miR-137 at endogenous levels, the RIP assay was carried out in KHOS/DXR and U2OS/DXR cells. As presented in Figure 3(g), circPVT1 and miR-137 were obviously enriched in Ago2 pellets of KHOS/DXR and U2OS/DXR cell extracts when compared with the IgG control group. Collectively, these data suggested that circPVT1 could directly bind with miR-137.

### 3.4. circPVT1 Silencing Enhanced DXR Sensitivity in DXR-Resistant Osteosarcoma Cells by Targeting miR-137

As mentioned above, circPVT1 played an important role in DXR resistance of osteosarcoma cells, and miR-137 served as a target of circPVT1. Hence, to explore whether circPVT1 could regulate DXR resistance of osteosarcoma cells by targeting miR-137, we performed the rescue experiments. As shown in Figure 4(a), the knockdown of circPVT1 promoted the expression level of miR-137, while the introduction of miR-137 inhibitor abated the effect on KHOS/DXR and U2OS/DXR cells. Moreover, IC50 determination indicated that circPVT1 silencing notably reduced DXR resistance in KHOS/DXR and U2OS/DXR cells, which was abolished by the downregulation of miR-137 (Figure 4(b)). Also, miR-137 inhibitor strikingly abrogated si-circ-triggered reduction in the number of colonies and enhancement in the apoptosis rate in KHOS/DXR and U2OS/DXR cells (Figures 4(c) and 4(d)). In addition, western blot results suggested that the inhibition of Bcl-2, ABCB1, and MRP-1 and the promotion of c-caspase-3 due to the circPVT1 knockdown were reversed by miR-137 inhibitor in KHOS/DXR and U2OS/DXR cells (Figure 4(e)). All of these results suggested that the downregulation of miR-137 could partly abolish the circPVT1-silencing-induced DXR sensitivity in DXR-resistant osteosarcoma cells.

### 3.5. TRIAP1 Was a Target of miR-137

It has been reported that TRIAP1 was related to drug chemosensitivity in osteosarcoma cells. So, the expression level of TRIAP1 was examined in osteosarcoma. RT-qPCR and western blot analysis verified that TRIAP1 was increased in the osteosarcoma tissues and the chemoresistant group relative to their respective controls (Figures 5(a)–5(d)). Meanwhile, we further proved that both mRNA level and protein level of TRIAP1 were distinctly upregulated in the DXR-resistant osteosarcoma cells (KHOS/DXR and U2OS/DXR) in comparison with other cells (Figures 5(e) and 5(f)). Interestingly, there was a negative correlation between TRIAP1 and miR-137 in osteosarcoma tissues (Figure 5(g)). As widely believed, miRNAs could exert the function by interacting with the target genes. By using bioinformatic software starbase 3.0, TRIAP1 was found to have some complementary base pairing with miR-137 (Figure 5(h)). Then, the latent binding was detected in 293T cells through a dual-luciferase reporter assay. Results suggested that the exogenetic expression of miR-137 prominently repressed the luciferase activity of TRIAP1 3′UTR wt reporter plasmid but not that of TRIAP1 3′UTR mut reporter plasmid (Figure 5(i)). Consistent with bioinformatic analysis and luciferase assay, the RIP assay indicated that the levels of miR-137 and TRIAP1 were specifically enriched in the anti-Ago2 group compared with the anti-IgG group in KHOS/DXR and U2OS/DXR cells (Figure 5(j)). Besides, the transfection efficiency of miR-137 mimic was detected in KHOS/DXR and U2OS/DXR cells. As exhibited in Figure 5(k), compared with cells transfected with mimic NC, the miR-137 level was evidently increased in miR-137 mimic-transfected KHOS/DXR and U2OS/DXR cells. All in all, miR-137 could interact with TRIAP1.

### 3.6. TRIAP1 Upregulation Partially Abrogated the Inductive Effect of miR-137 Improved on DXR Sensitivity in DXR-Resistant Osteosarcoma Cells

Next, we explored the regulatory role of miR-137 and TRIAP1 on DXR resistance in osteosarcoma cells. Firstly, the overexpression efficiency of oe-TRIAP1 was examined and shown in Figures 6(a) and 6(b). Then, the drug resistance assay suggested that the miR-137 mimic enhanced DXR sensitivity in KHOS/DXR and U2OS/DXR cells, while the reintroduction of oe-TRIAP1 mitigated these effects (Figure 6(c)). What is more, TRIAP1 overexpression attenuated the inhibitory effect of miR-137 mimic on the clone number in KHOS/DXR and U2OS/DXR cells (Figure 6(d)). Synchronously, oe-TRIAP1 abrogated the positive impact of miR-137 upregulation on the apoptosis rate in KHOS/DXR and U2OS/DXR cells (Figure 6(e)). Additionally, we further assessed the effect of miR-137 and TRIAP1 on the protein levels of Bcl-2, c-caspase-3, ABCB1, and MRP-1. Data indicated that the overexpression of TRIAP1 significantly reversed miR-137 mimic-caused decrease in Bcl-2, ABCB1, and MRP-1 and increase in c-caspase-3 in KHOS/DXR and U2OS/DXR cells (Figure 6(f)). Taken together, these results suggested that miR-137 could reinforce DXR sensitivity through modulating TRIAP1.

### 3.7. TRIAP1 Was Positivity Regulated by circPVT1/miR-137

Based on the above findings, we speculated that circPVT1 could exert the role through regulating the miR-137/TRIAP1 axis. Therefore, we used the rescue assays to verify the assumption. As presented in Figures 7(a) and 7(b), the knockdown of circPVT1 blocked the mRNA level and protein level of TRIAP1 in KHOS/DXR and U2OS/DXR cells; however, miR-137 inhibitor could reverse these effects. That was to say, circPVT1 could positively regulate TRIAP1 through sponging miR-137.

### 3.8. circPVT1 Knockdown Hindered Tumor Growth in Osteosarcoma Cells *In Vivo*

In addition, to confirm the functional effect of circPVT1 on tumor growth *in vivo*, a xenograft tumor mouse model was established. As shown in Figures 8(a) and 8(b), the tumor volume and tumor weight reduced in the presence of circPVT1 knockdown, implying that the silencing of circPVT1 could block osteosarcoma tumor growth *in vivo*. Furthermore, RT-qPCR assays indicated that the levels of circPVT1 and TRIAP1 were declined in tumor tissues from sh-circ-transfected KHOS/DXR cells, whereas the miR-137 level was enhanced (Figure 8(c)). Also, western blot results proved that the TRIAP1 protein level was remarkably lower in tumor tissues from the sh-circ group than the sh-NC group (Figure 8(d)). Meanwhile, the decreased protein levels of Bcl-2, ABCB1, and MRP-1 and increased c-caspase-3 level were observed in the sh-circ group versus the sh-NC group (Figure 8(e)). All of these data suggested that circPVT1 knockdown could inhibit tumor growth and improved drug sensitivity in osteosarcoma *in vivo*.

## 4. Discussion

Currently, it has been acknowledged that DXR is an effective chemotherapy drug for the treatment of osteosarcoma patients [30, 31], but drug resistance is becoming a predominant cause of failure. In recent years, the biological functions of circRNAs have been gradually identified due to the development of bioinformatic analysis and high-throughput sequencing [32–34]. In fact, some studies have confirmed that circRNAs are related to the development of chemotherapeutic resistance in human cancers, including osteosarcoma [35–37]. Noticeably, as a carcinogenic factor, a higher circPVT1 expression level has been exhibited in osteosarcoma cell lines [13, 38]. Furthermore, a recent document presented that the upregulation of circPVT1 expedited the resistance of osteosarcoma cells to DXR [14]. Yet, the potential mechanism of circPVT1 in DXR-resistant osteosarcoma is still unclear.

In this paper, circPVT1 was presented to exert high expression in DXR-resistant osteosarcoma tissues and cell lines, consistent with earlier studies [14]. Also, as an ATP-binding cassette member, ABCB1 known as P-glycoprotein (P-gp) has been identified as one of the important mechanisms of drug resistance through boosting the efflux of chemotherapeutic drugs from cancer cells [39–41]. Multidrug resistance-associated protein 1 (MRP-1/ABCC1), a member of the ATP-binding cassette, produced multidrug resistance by actively exporting antitumor drugs clinically [42, 43]. In this study, the high expression of ABCB1 and MRP-1 was viewed in DXR-resistant osteosarcoma tissues and cell lines, confirming the drug resistance of osteosarcoma tissues and cells. Functionally, circPVT1 deficiency enhanced DXR sensitivity, curbed DXR-caused cell proliferation, and facilitated DXR-triggered apoptosis in DXR-resistant osteosarcoma cells *in vitro*. More importantly, our results verified that the knockdown of circPVT1 could block ABCB1 and MRP-1 levels in DXR-resistant osteosarcoma cells, implying that circPVT1 silencing might mitigate the drug resistance of osteosarcoma cells. Apart from that, the drug resistance of circPVT1 was also verified in osteosarcoma *in vivo*.

Recently, one hypothesis is that circRNAs could exert their effects through serving as a sponge for miRNAs [44]. In this paper, we found that miR-137 was expressed at a low level in DXR-resistant osteosarcoma tissues and cell lines, in agreement with some previous reports [22]. In osteosarcoma tissues, we found a negative correlation between circPVT1 and miR-137. Therefore, using the online-based bioinformatic software starbase 3.0, we observed that miR-137 could interact with circPVT1, as demonstrated by dual-luciferase reporter and RIP assays. Functional analysis presented that the knockdown of miR-137 could partly abrogate the circPVT1 silencing-triggered improvement in DXR sensitivity. In accordance with our data, the inductive impact of miR-137 on DXR sensitivity was confirmed in breast cancer [45] and neuroblastoma [46].

Up to now, it has been confirmed that miRNAs could exert the role by the interaction with their target genes [47]. In the manuscript, an apparent increase of TRIAP1 was viewed in DXR-resistant osteosarcoma tissues and cell lines. Also, the TRIAP1 level was inversely related to miR-137 in osteosarcoma tissues. A prior study has pointed out that TRIAP1 was implicated in chemosensitivity in osteosarcoma [26]. Hence, TRIAP1 was chosen for in-depth investigations. In the paper, our results confirmed that TRIAP1, as a direct target of miR-137, partly reversed the promotion effect of miR-137 overexpression on DXR sensitivity. In addition, mechanistic analysis verified that miR-137 inhibitor could partly overturn the suppression effect of circPVT1 silencing on the TRIAP1 level in DXR-resistant osteosarcoma cells, validating that circPVT1 could function as a sponge of miR-137 to upregulate TRIAP1 expression.

## 5. Conclusion

Our findings first proved that the regulatory role of circPVT1 in DXR resistance of osteosarcoma was mediated by the miR-137/TRIAP1 axis, providing an underlying circRNA-targeted therapy for osteosarcoma.

## Figures and Tables

**Figure 1:** circPVT1 was elevated in osteosarcoma tissues and cells. (a) RT-qPCR assay was employed to detect the expression level of circPVT1 in osteosarcoma tissues (*n* = 52) and normal tissues (*n* = 45). (b) circPVT1 level was measured in the chemosensitive group (31) and the chemoresistant group (21). (c) Western blot assay was used to measure the protein levels of ABCB1 and MRP-1 in 52 osteosarcoma tissues and 45 normal tissues. (d) ABCB1 and MRP-1 protein levels were assessed in the chemosensitive group (*n* = 31) and the chemoresistant group (*n* = 21). (e) Relative circPVT1 expression was examined in the human fetal osteoblastic cell line (hFOB1.19), parental osteosarcoma cells (KHOS and U2OS), and DXR-resistant osteosarcoma cells (KHOS/DXR and U2OS/DXR). (f) The protein levels of ABCB1 and MRP-1 were detected in parental osteosarcoma cells (KHOS and U2OS) and DXR-resistant osteosarcoma cells (KHOS/DXR and U2OS/DXR). ^∗^*P* < 0.05.

**Figure 2:** circPVT1 knockdown-sensitized KHOS/DXR and U2OS/DXR cells to DXR. KHOS/DXR and U2OS/DXR cells were transfected with si-NC and si-circ. (a) circPVT1 level was measured in transfected KHOS/DXR and U2OS/DXR cells. (b) CCK-8 assay was applied to detect the viability and IC50 value in transfected KHOS/DXR and U2OS/DXR when exposed to DXR. (c) Cell colony formation assay was performed to measure the clone number in transfected KHOS/DXR and U2OS/DXR cells. (d) Flow cytometry assay was conducted to examine the apoptosis rate in transfected KHOS/DXR and U2OS/DXR cells. (e) The protein levels of Bcl-2, c-caspase-3, ABCB1, and MRP-1 were evaluated in transfected KHOS/DXR and U2OS/DXR cells. ^∗^*P* < 0.05.

**Figure 3:** miR-137 was a direct target of circPVT1. (a, b) Relative miR-137 expression was detected in osteosarcoma tissues (*n* = 52), normal tissues (*n* = 45), chemosensitive group (*n* = 31), and chemoresistant group (*n* = 21). (c) miR-137 level was assessed in hFOB1.19, KHOS, KHOS/DXR, U2OS, and U2OS/DXR cells. (d) The expression correlation between miR-137 and circPVT1 in osteosarcoma tissues was analyzed by Pearson correlation analysis. (e) The binding sites between circPVT1 and miR-137 were predicted by using starbase 3.0. (f) The potential binding relationship between circPVT1 and miR-137 in 293T cells was verified by the dual-luciferase reporter assay. (G) RIP assay was conducted in KHOS/DXR and U2OS/DXR cell extracts to detect miR-137 endogenously associated with circPVT1. ^∗^*P* < 0.05.

**Figure 4:** circPVT1 silencing enhanced DXR sensitivity in DXR-resistant osteosarcoma cells by the upregulation of miR-137. KHOS/DXR and U2OS/DXR cells were transfected with si-NC and si-circ, si-circ+inhibitor NC, and si-circ+miR-137 inhibitor. (a) Relative miR-137 expression was detected in transfected KHOS/DXR and U2OS/DXR cells. (b) Cell viability and IC50 value were assessed in transfected KHOS/DXR and U2OS/DXR cells. (c) The clone number was calculated in transfected KHOS/DXR and U2OS/DXR cells. (d) Apoptosis rate was measured in transfected KHOS/DXR and U2OS/DXR cells. (e) The protein levels of Bcl-2, c-caspase-3, ABCB1, and MRP-1 were examined in transfected KHOS/DXR and U2OS/DXR cells. ^∗^*P* < 0.05.

**Figure 5:** TRIAP1 served as a target of miR-137. (a, b) Relative TRIAP1 mRNA expression was examined in 52 osteosarcoma tissues, 45 normal tissues, chemosensitive group (31), and chemoresistant group (21). (c, d) TRIAP1 protein levels were assessed in 52 osteosarcoma tissues, 45 normal tissues, chemosensitive group (31), and chemoresistant group (21). (e, f) Both mRNA level and protein level of TRIAP1 were measured in hFOB1.19, KHOS, KHOS/DXR, U2OS, and U2OS/DXR cells. (g) Pearson correlation analysis was applied to assess the expression association between TRIAP1 and miR-137 in osteosarcoma tissues. (h) The binding sites between miR-137 and TRIAP1 3′UTR wt and the sequences of TRIAP1 3′UTR mut. (i) Dual-luciferase reporter assay was used to prove the potential binding relationship between miR-137 and TRIAP1 in 293T cells. (j) The interaction between miR-137 and TRIAP1 3′UTR in KHOS/DXR and U2OS/DXR cells was confirmed by using the RIP assay. (k) miR-137 level was detected in KHOS/DXR and U2OS/DXR cells transfected with mimic NC and miR-137 mimic. ^∗^*P* < 0.05.

**Figure 6:** miR-137 improved DXR sensitivity in DXR-resistant osteosarcoma cells by targeting TRIAP1. (a, b) The mRNA level and protein level of TRIAP1 were detected in KHOS/DXR and U2OS/DXR cells transfected with vector and oe-TRIAP1. (c–g) KHOS/DXR and U2OS/DXR cells were transfected with mimic NC, miR-137 mimic, miR-137 mimic+vector, and miR-137 mimic+oe-TRIAP1. (c) Cell viability was measured in transfected KHOS/DXR and U2OS/DXR cells. (d) The clone number was examined in transfected KHOS/DXR and U2OS/DXR cells. (e) Apoptosis rate was detected in transfected KHOS/DXR and U2OS/DXR cells. (f) The protein levels of Bcl-2, c-caspase-3, ABCB1, and MRP-1 were assessed in transfected KHOS/DXR and U2OS/DXR cells. ^∗^*P* < 0.05.

**Figure 7:** circPVT1 modulated TRIAP1 expression by sponging miR-137. KHOS/DXR and U2OS/DXR cells were transfected with si-NC, si-circ, si-circ+inhibitor NC, and si-circ+miR-137 inhibitor. (a, b) The mRNA level and protein level of TRIAP1 were detected in transfected KHOS/DXR and U2OS/DXR cells. ^∗^*P* < 0.05.

**Figure 8:** circPVT1 knockdown inhibited tumor growth in osteosarcoma cells *in vivo.* (a, b) Tumor volume and tumor weight were detected in xenografts. (c) The levels of circPVT1, miR-137, and TRIAP1 in xenografts were assessed by RT-qPCR assay. (d) TRIAP1 protein level was measured in xenografts by western blot assay. (e) The protein levels of Bcl-2, c-caspase-3, ABCB1, and MRP-1 were examined in xenografts. ^∗^*P* < 0.05.

**Table 1:** The sequences of primers for RT-PCR used in this study.

Names	Sequences (5′-3′)
circPVT1: forward	AGTCCGCTGTCACCTTGAAT
circPVT1: reverse	TGGCACAACCACTGCTTTTA
miR-137: forward	ATTGCTTAAGAATACGCGT
miR-137: reverse	GAACATGTCTGCGTATCTC
TRIAP1: forward	AGGATTTCGCAAGTCCAGAA
TRIAP1: reverse	GCTGATTCCACCCAAGTAT
U6: forward	CTCGCTTCGGCAGCACA
U6: reverse	AACGCTTCACGAATTTGCGT
GAPDH: forward	GTGGACCTGACCTGCCGTCT
GAPDH: reverse	GGAGGAGTGGGTGTCGCTGT

## Data Availability

Please contact the correspondence author for the data request.
